The article "Systematic evaluation of percutaneous radiofrequency ablation versus percutaneous ethanol injection for the treatment of small hepatocellular carcinoma: a meta-analysis" was retracted in 2015. Reason: compromised peer review.

# Systematic evaluation of percutaneous radiofrequency ablation versus percutaneous ethanol injection for the treatment of small hepatocellular carcinoma: a meta-analysis

**DOI:** 10.1186/2047-783X-19-39

**Published:** 2014-08-20

**Authors:** Rong-Hua Xu, Wei Gao, Chao Wang, De-Kai Guo, Lin Tang, Hui Zhang, Cong-Jun Wang

**Affiliations:** 1 Department of Oncology Surgery, the Affiliated Hospital of Hainan Medical College, 31 Longhua Road, Haikou 570102, Hainan Province, China; 2 Department of Hepatobiliary and Pancreatic Diseases, Shanghai East Hospital, Tongji University School of Medicine, 150 Jimo Road, Pudong New District, Shanghai 200120, China; 3 Departments of Surgery, University of Michigan Medical School, 1500 E Medical Center Dr, Ann Arbor 48105, Michigan, USA; 4 Translational Oncology Program, University of Michigan Medical School, 1600 Huron Parkway, Ann Arbor MI 48109, Michigan, USA

**Keywords:** percutaneous radiofrequency ablation, percutaneous ethanol injection, small hepatocellular carcinoma, system evaluation, meta-analysis

## Abstract

**Background:**

Radiofrequency ablation (RFA) and percutaneous ethanol injection (PEI) have been used for patients with hepatocellular carcinoma (HCC). However, which therapy is superior remains to be further elucidated. We aimed to conduct a systematic review to assess survival and local tumor recurrence rate with RFA compared with PEI therapy for HCC.

**Methods:**

We conducted systematic review and meta-analysis of randomized controlled trials (RCTs) published up to 2014 in PubMed, MEDLINE, EMBASE, EBSCO, Springer, Ovid and the Cochrane library. Only RCTs that evaluated survival rate and occurrence of HCC between RFA and PEI therapy were included. The OR (odds ratio) with a 95% confidence interval (CI) was calculated by the Revman 5.0 software.

**Results:**

A total of six studies including 983 HCC patients were eligible for this analysis. The survival rate showed a significant benefit under RFA therapy over PEI at 1-year (*P* = 0.02, OR = 1.88, 95% CI: 1.09 to 3.22), 2-years (*P* = 0.0003, OR = 2.06, 95% CI: 1.39 to 3.05) and 3-years (*P* = 0.0007, OR = 1.68, 95% CI: 1.25 to 2.27). Likewise, RFA achieved significantly lower rates of local tumor recurrence over PEI at 1-year (*P* = 0.002, OR = 0.43, 95% CI: 0.26 to 0.73), 2-year (*P* = 0.03, OR = 0.33, 95% CI: 0.12 to 0.88) and 3-year (*P* = 0.003, OR = 0.61, 95% CI: 0.43 to 0.84).

**Conclusions:**

The current evidence suggests that RFA is superior to PEI in better survival and local disease control for small HCCs <5 cm in diameter and that RFA is worthy of promotion in clinical applications.

## Background

Hepatocellular carcinoma (HCC) is the sixth leading tumor in the world [1], and it is estimated that its incidence will continue to rise in coming decades [2,3]. Approximately 80% to 90% of primary HCC is accompanied by cirrhosis, which works together with HCC leading to liver failure [4]. The pathogenesis for HCC is rather complicated since many risk factors are involved.

At present, liver resection and transplantation can improve the survival rate of HCC, but long waiting time due to the shortage of donor organs may result in tumor progression. Given these limitations, many nonsurgical methods have been proposed, including percutaneous ethanol injection (PEI), radiofrequency ablation (RFA), microwave thermal ablation and percutaneous acid injection. Among them, RFA is a localized thermal treatment technique designed to produce tumor destruction by heating tumor tissue to a temperature exceeding 50°C [5]. With the development of this technique, RFA has recently gained greater interest and become the most widely applied liver-directed treatment technique [6,7]. In recent years, several studies concerning the comparisons between therapies of RFA and PEI for HCC have been published [8-10]. However, most of them did not involve a comprehensive analysis of survival rate and occurrence of HCC in patients undergoing RFA and PEI therapy. Although the meta-analysis of Bouza *et al*. has analyzed survival rate and occurrence rate of HCC with the two therapies, the sample size was relatively small. In addition, the included studies in their meta-analysis did not contain the latest studies on RFA [11].

Therefore, we conducted this study and aimed to perform a further systematic assessment on the efficacy of treatment with percutaneous RFA and PEI on survival and recurrence rates in patients with HCCs <5 cm in diameter (1 to 3 nodules).

## Methods

### Literature search

A review of the literature was conducted in MEDLINE, EMBASE, EBSCO, Springer, Ovid and the Cochrane library up to 2014 using the following key words: ‘hepatocellular carcinoma’ AND ‘HCC’ AND ‘radiofrequency ablation’ AND ‘ethanol/alcohol injection’ with language limited to English.

### Inclusion criteria

To be eligible for this analysis, published articles had to meet the following criteria: 1) all the patients were confirmed as HCC by pathological diagnosis and computed tomography (CT) or magnetic resonance imaging (MRI) diagnosis; 2) none of the patients had received any anticancer treatments before; 3) all studies were randomized controlled trials (RCTs)conducted on more than ten adults; 4) tumor diameter was not more than 5 cm and lesion number was 1 to 3; and 5) all the results from the studies were required to describe data related to at least one of the following assessment indexes: 1-, 2- and 3-year-survival rates or 1-, 2- and 3-year local tumor recurrence rate.

### Quality assessment

The Cochrane Handbook for Systematic Reviews of Interventions (http://handbook.cochrane.org) [12] was used to evaluate the quality of the included studies independently by two investigators. Any disagreement was subsequently resolved by discussion with another investigator.

### Data extraction

Two investigators independently extracted the following data from original publications: 1) general information including subject, authors, publication year and source of the research; 2) details of the study design and duration of follow-up; and 3) the experimental results of efficacy including survival and recurrence rate. Software Engauge Digitizer 4.1 (Geeknet, Inc., Mountain View, California, US, http://digitizer. Sourceforge.net) was utilized to extract data from survival curve as necessary.

### Statistical analysis

Revman 5.0 (Cochrane Collaboration, Oxford, UK), which was provided by the Cochrane Collaboration, was used for meta-analysis and forest plot. The results were presented as pooled odds ratio (OR) and 95% confidence interval (CI). Chi-square and I^2^ test were performed to determine the heterogeneity among studies. If no significant heterogeneity was indicated (*P* >0.05, I^2^ <50%), a fixed effects model was used in analysis. Otherwise (*P* <0.05, I^2^ >50%), a random effects model was selected.

## Results

### Literature selection

A total of 2,876 titles were retrieved (276 from MEDLINE, 528 from EMBASE, 202 from EBSCO, 867 from Springer, 984 from Ovid and 19 from the Cochrane library). Under the inclusion criteria, six studies including 983 HCC patients were selected [8-10,13-15]. Among them, only three studies provided all the assessment indexes [8,9,14], one study lacked a 2-year survival rate and a 2-year local tumor recurrence rate [13], and one lacked a 3-year survival rate and a 3-year local tumor recurrence rate [15]. Furthermore, one study did not describe the 2-year local tumor recurrence rate [10]. All these studies adopted a random method and allocation concealment program, but no one mentioned whether or not a double-blind method was used. The procedure for literature selection was presented in Figure 1.

**Figure 1:** The flow chart of literature search and selection.

### Survival rate

In our study, all of the six included studies assessed 1-year survival rate [8-10,13-15], five studies assessed a 2-year survival rate [8-10,14,15], and five studies assessed a 3-year survival rate [8-10,13,14] of patients treated with two types of therapies. The fixed effects model was used to analyze the differences between two therapies on survival rates for the absence of apparent heterogeneity (*P* >0.05, I^2^ <50%). Our results showed that patients treated with RFA obtained a significantly higher survival benefit in 1-year (*P* = 0.02, OR = 1.88, 95% CI: 1.09 to 3.22) (Figure 2A), 2-year (*P* = 0.0003, OR = 2.06, 95% CI: 1.39 to 3.05) (Figure 2B) and 3-year survival rate (*P* = 0.0007, OR = 1.68, 95% CI: 1.25 to 2.27) (Figure 2C) than those treated with PEI.

**Figure 2:** **The survival rates evaluation between percutaneous radiofrequency ablation (RFA) and percutaneous ethanol injection (PEI) therapies. A**) 1-year survival rate; **B**) 2-year survival rate; **C**) 3-year survival rate. CI, confidence interval; OR, odds radio. RFA, radiofrequency ablation; PEI, percutaneous ethanol injection.

### Local tumor recurrence rate

In this meta-analysis, there was no apparent heterogeneity in 1-year (*P* = 0.57, I^2^ <50%) and 3-year (*P* = 0.60, I^2^ <50%) local tumor recurrence rate. On the contrary, significant heterogeneity was presented in 2-year local tumor recurrence rate (*P* = 0.01, I^2^ >50%). Therefore, the fixed effects model was selected for 1- and 3-year local tumor recurrence rate, while the random effects model was applied to the 2-year rate. Further analysis suggested that all the studies reported 1-year tumor recurrence rate, up to four of the six studies assessed 2-year local tumor recurrence rate [8,9,14,15] and five studies described 3-year local tumor recurrence rate [8-10,13,14]. The results indicated that the 1-year (*P* = 0.002, OR = 0.43, 95% CI: 0.26 to 0.73) (Figure 3A), 2-year (*P* = 0.03, OR = 0.33, 95% CI: 0.12 to 0.88) (Figure 3B) and 3-year (*P* = 0.003, OR = 0.61, 95% CI: 0.43 to 0.84) (Figure 3C) local tumor recurrence rate of HCC treated with RFA was significantly lower than that with PEI.

**Figure 3:** **The local tumor recurrence rates evaluation between percutaneous radiofrequency ablation (RFA) and percutaneous ethanol injection (PEI) therapies. A**) 1-year local tumor recurrence rate; **B**) 2-year local tumor recurrence rate; **C**) 3-year local tumor recurrence rate. CI, confidence interval; OR, odds radio. RFA, radiofrequency ablation; PEI, percutaneous ethanol injection.

## Discussion

At present, RFA and PEI are verified to be feasible and of benefit in non-operable patients and are used as bridging therapies before liver transplantation [16,17]. In recent years, many studies have demonstrated that RFA is superior to PEI in efficacy and safety for the management of HCC [13,18]. However, only a small fraction of these studies were relevant to survival rate and tumor recurrence rate [11]. Therefore, we performed this meta-analysis to evaluate the efficacy of RFA and PEI for the treatment of HCC patients by comparing their effects in survival rates and local tumor recurrence rates.

In the present meta-analysis, a total of six studies were selected in our analysis [8-10,13-15]. Our results showed that treatment with RFA achieved higher survival rates at 1, 2, and 3 years than treatment with PEI. In addition, we further evaluated the local tumor recurrence rate, and the results showed that treatment with RFA had a lower risk of local tumor recurrence at 1, 2, and 3years compared with PEI.

As far as we know, RFA was applied to the management of HCC when the recurrent tumor was <6 cm in diameter or when there were three or fewer tumor nodules [19]. In contrast, PEI therapy is considered to be effective for the treatment of HCC of relatively small size (less than 1 cm of necrosis) [20]. Due to this, RFA covers a larger area in the treatment for HCC. Consistent with this conclusion, the results of Shen A *et al*. demonstrated that RFA appears superior to PEI in local tumor control for small HCCs <3 cm in diameter [21]. In our meta-analysis, the tumor sizes in the six studies were all less than 5 cm in diameter. The higher survival rates under RAF therapy compared with PEI, as indicated by our results, can also be explained by the fact that RFA has greater complete radiological tumor response [22,23]. Moreover, tumor recurrence after RFA carries significant prognostic value in relation to overall survival [24]. Related studies have indicated that RFA can significantly lower local tumor recurrence rates [25,26], which is consistent with our results.

However, the following limitations of our meta-analysis should be considered. First, the magnitude of included studies and participants was relatively small. Second, all of the included studies lacked of long-term data on patient survival, and most of them have follow-up periods of approximately 2 to 3 years. Third, these studies are limited to RCTs published in English, which may have brought in publication bias. Fourth, a small proportion of data were directly extracted from the survival curves and local tumor recurrence curves without raw data, which may reduce the accuracy of these data. In addition, there was a shortage of subgroup analysis that may contribute to 2-year local tumor recurrence rate. Therefore, future studies should take tumor size, specific site of the tumor and other subgroup effects into consideration.

## Conclusions

Based on this analysis, we conclude that RFA is more advantageous than PEI therapy for HCC management with respect to survival rate and local tumor recurrence rate, and deserves to be applied to clinical practice. Nevertheless, due to the limitations in our meta-analysis as presented above, further validation regarding different sizes of tumor therapy should be obtained in more randomized studies comparing RFA and PEI.

## Abbreviations

CI: confidence interval; CT: computed tomography; HCC: hepatocellular carcinoma; MRI: magnetic resonance imaging; OR: odds ratio; PEI: percutaneous ethanol injection; RCT: randomized controlled trial; RFA: radiofrequency ablation.

## Competing interests

The authors declare that they have no competing interests.

## Authors’ contributions

RHX and WG participated in the design of this study, and they both performed the statistical analysis. CW carried out the study together with DKG and LT. HZ and CJW drafted the manuscript. All authors read and approved the final manuscript.
